# Research on AR-AKF Model Denoising of the EMG Signal

**DOI:** 10.1155/2021/9409560

**Published:** 2021-11-08

**Authors:** Sijia Chen, Zhizeng Luo, Tong Hua

**Affiliations:** Institute of Intelligent Control and Robotics Hangzhou Dianzi University, Hangzhou 310018, China

## Abstract

Electromyography (EMG) signals can be used for clinical diagnosis and biomedical applications. It is very important to reduce noise and to acquire accurate signals for the usage of the EMG signals in biomedical engineering. Since EMG signal noise has the time-varying and random characteristics, the present study proposes an adaptive Kalman filter (AKF) denoising method based on an autoregressive (AR) model. The AR model is built by applying the EMG signal, and the relevant parameters are integrated to find the state space model required to optimally estimate AKF, eliminate the noise in the EMG signal, and restore the damaged EMG signal. To be specific, AR autoregressive dynamic modeling and repair for distorted signals are affected by noise, and AKF adaptively can filter time-varying noise. The denoising method based on the self-learning mechanism of AKF exhibits certain capabilities to achieve signal tracking and adaptive filtering. It is capable of adaptively regulating the model parameters in the absence of any prior statistical knowledge regarding the signal and noise, which is aimed at achieving a stable denoising effect. By comparatively analyzing the denoising effects exerted by different methods, the EMG signal denoising method based on the AR-AKF model is demonstrated to exhibit obvious advantages.

## 1. Introduction

Surface electromyography (sEMG) refers to a weak bioelectric signal recorded by surface electromyography pick-up electrodes, which is capable of reflecting information associated with muscle and bone activity [1]. It has been extensively employed in sports medicine and rehabilitation training, and it is an ideal control signal for artificial prostheses and bionic control [2, 3].

sEMG is recognized as a nonlinear and nonstationary signal. The useful signal displays the major distribution between 10 Hz and 500 Hz, which is extremely weak (with the amplitude of only *μ*V level). The signal is vulnerable to a range of characteristics (e.g., interference, time variance, and randomness) [4]. The sEMG signal is collected by detecting electrodes placed on the skin surface, and such a collecting process is easy to be affected by surrounding environments. On the whole, sEMG noise sources consist of inherent noise of electronic devices, environmental noise, noise generated by electrode jitter and micromovement, and interference noise created by other human bioelectric signals. In addition, the signal-to-noise ratio (SNR) of the sEMG signal decreases with the increase in the muscle contraction force. The mentioned noises may seriously affect the quality of the signal and may even fail to effectively achieve the detection and analysis applications. Accordingly, noise removal processing should be performed before sEMG is studied in depth.

On the hardware, noise interference can be suppressed by taking shielding and grounding or introducing high- and low-pass filters, as well as notch filters, which is recognized as a routine operation. However, the noise interference of the sEMG cannot be eliminated through hardware processing independently [5] . As digital signal processing technologies are leaping forward, digital filtering has become a vital approach to reduce noise interference. The common existing sEMG signal denoising methods comprise wavelet denoising [6, 7], empirical mode decomposition (EMD) [8, 9], adaptive filtering [10], and principal component analysis (PCA) [11] and independent component analysis (ICA) [12]. These denoising methods exhibit their own advantages and disadvantages, and a balance remains difficult to reach between denoising and muscle power signal restoration. Even in a segment of signal, there may be varied levels of noise, and it is difficult to perform well in different levels of noise.

An autoregressive (AR) model is a prediction model that creates a linear sum of previous data. The coefficients of the AR model are used in sEMG classification [13, 14]. The AR model of order is usually according to the previous works; then, the model is determined. There is no way to judge whether the AR model is appropriate for sEMG data. In order to overcome existing problems above, we propose the following method.

The AR-AKF model-based denoising method organically combines the dynamic modeling ability of the autoregressive model and the time-varying noise estimation ability of the adaptive Kalman filter. By using AKF, the noise in the sEMG is effectively eliminated. Moreover, with the AR model, the signal affected by noise can be restored. This method is capable of learning and tracking, as well as regulating model parameters by complying with the adaptive criteria in the absence of any prior statistical knowledge regarding the signal and noise, as an attempt to achieve a stable denoising effect. Theoretically, this method exhibits better applicability, which is also suitable for other similar bioelectric signals.

## 2. AR-AKF Model

Set *x*_*t*_ as the EMG signal at sampling time *t*, and *x*_*t*−*n*_ signifies the EMG signal at sampling time *t* − *n*, which is a random noise. Moreover, an *n*-order AR model can be adopted to express the EMG signal. An *n*-order AR model of sEMG, written as AR(*n*), is

(1) $$\begin{array}{c} x_{t}=\Phi_{1}x_{t-1}+\Phi_{2}x_{t-2}+\cdots +\Phi_{n}x_{t-n}+\varepsilon_{t}, \end{array}$$

where *n* denotes the model order, *ϕ*_*n*_ represents the model parameter, and *ε*_*t*_ is the white noise with zero mean and variance *σ*_*ε*_^2^.

The main work for AR(*n*) model building is to estimate the values of parameters *n*, *ϕ*_1_, *ϕ*_2_ ⋯ , *ϕ*_*n*_, and *ε*_*t*_ in the model. The reason is that *ϕ*_1_, *ϕ*_2_ ⋯ , *ϕ*_*n*_ and *ε*_*t*_ satisfy

(2) $$\begin{array}{c} \varepsilon_{t}=x_{t}-\phi_{1}x_{t-1}-\phi_{2}x_{t-2}-\cdots +\phi_{n}x_{t-n}, \end{array}$$

(3) $$\begin{array}{c} {\sigma_{\varepsilon }}^{2}=\frac{1}{N-n}\overset{N}{\underset{t=n+1}{\sum }}{\left(x_{t}-\overset{n}{\underset{i=1}{\sum }}\varphi_{i}x_{t-i}\right)}^{2}, \end{array}$$

where *N* denotes the number of samples.

Thus, if *ϕ*_1_ is estimated, *σ*_*ε*_^2^ can be estimated by equation (3).

The method of parameter estimation falls to direct and indirect methods. Direct methods comprise the least square method, Yule-Walker equation method, Ulrych-Clayton method, etc. In addition, indirect methods include the LUD method, BSMF method, and Burg method. Using the least square method to estimate the parameters is considered to be extremely simple. The parameter estimation is unbiased with high accuracy, as expressed by

(4) $$\begin{array}{c} Y=X\phi +\varepsilon , \end{array}$$

where *Y* = [*x*_*n*+1_ *x*_*n*+2_  ⋯  *x*_*N*_]^*T*^, $\phi ={\left[\begin{array}{cccc} \phi_{1} & \phi_{2} & \cdots & \phi_{n} \end{array}\right]}^{T}$, and $\varepsilon ={\left[\begin{array}{cccc} \varepsilon_{n+1} & \varepsilon_{n+2} & \cdots & \varepsilon_{N} \end{array}\right]}^{T}$.

Subsequently, the least square estimate of *ϕ* is

(5) $$\begin{array}{c} \phi ={\left(X^{T}X\right)}^{-1}X^{T}Y. \end{array}$$

The model order *n* can be determined by complying with the applicability test criterion of the model. Common information criteria consist of FPE (Final Prediction Error), AIC (An Information Criterion), and BIC (Bayesian Information Criterion) criteria of the Akaike information inspection criterion [13].

AIC function:

(6) $$\begin{array}{c} \text{AIC}\left(n\right)=N\ln\sigma_{\varepsilon }^{2}+2n. \end{array}$$

BIC function:

(7) $$\begin{array}{c} \text{BIC}\left(n\right)=N\ln\sigma_{\varepsilon }^{2}+n\ln N. \end{array}$$

FPE function:

(8) $$\begin{array}{c} \text{FPE}\left(n\right)=\frac{N+n}{N-n}\sigma_{\varepsilon }^{2}, \end{array}$$

where AIC(n), BIC(*n*), and FPE(*n*) represent the corresponding criterion indexes in the case of order *n*.

The model when the minimum value of the respective criterion function is selected is the applicable model. Thus, the estimation criterion of the optimal *n*-order is presented as

(9) $$\begin{array}{c} n^{*}=\underset{n}{\arg\min}\left\{\text{AIC}\left(n\right),\text{BIC}\left(n\right),\text{FPE}\left(n\right)\right\}. \end{array}$$

The core idea here is to simulate the volatility of the EMG signal through the AR(*n*) model and subsequently use adaptive filtering to correct the error attributed to random noise. To be suitable for adaptive filters, an accurate mathematical model is required. First, equation (1) is extended to *n* AR model groups of order 1 to *n*:

(10) $$\begin{array}{c} \begin{array}{c} x_{1}\left(t+1\right)=\Phi_{11}x_{1}\left(t\right)+\varepsilon_{1}\omega \left(t\right),\\ x_{2}\left(t+1\right)=\Phi_{21}x_{1}\left(t\right)+\Phi_{22}x_{2}\left(t\right)+\varepsilon_{2}\omega \left(t\right),\\ \cdots \\ x_{n}\left(t+1\right)=\Phi_{n1}x_{1}+\Phi_{n2}x_{2}\left(t\right)+\cdots +\Phi_{nn}x_{n}\left(t\right)+\varepsilon_{n}\omega \left(t\right). \end{array} \end{array}$$

Next, this model group is converted into an *n*-dimensional state space model:

(11) $$\begin{array}{c} \left[\begin{array}{c} x_{1}\left(t+1\right)\\ x_{2}\left(t+1\right)\\ \vdots \\ x_{n}\left(t+1\right) \end{array}\right]=\left[\begin{array}{cccc} \Phi_{11} & 0 & \cdots & 0\\ \Phi_{21} & \Phi_{22} & \cdots & 0\\ \vdots & \vdots & \ddots & \vdots \\ \Phi_{n1} & \Phi_{n2} & \cdots & \Phi_{nn} \end{array}\right]\left[\begin{array}{c} x_{1}\left(t\right)\\ x_{2}\left(t\right)\\ \vdots \\ x_{n}\left(t\right) \end{array}\right]+\left[\begin{array}{c} \varepsilon_{1}\\ \varepsilon_{2}\\ \vdots \\ \varepsilon_{n} \end{array}\right]\omega \left(t\right), \end{array}$$

(12) $$\begin{array}{c} z_{t}=\left[\begin{array}{cccc} \phi_{nl}, & \phi_{n2}, & \cdots & \phi_{nn} \end{array}\right]\left[\begin{array}{c} x_{t-1}\\ x_{t-2}\\ \vdots \\ x_{t-n} \end{array}\right]+\varepsilon_{t}, \end{array}$$

where (11) expresses the state transition equation, (12) presents the observation equation, *x* represents the measured EMG signal, *y* denotes the EMG observation signal, and *ϕ*_*ni*_ is the *i*-th parameter of the *n*-order AR model. The mentioned (11) and (12) can be simplified to the state space model below:

(13) $$\begin{array}{c} \left\{\begin{array}{c} X\left(t+1\right)=AX\left(t\right)+w\left(t\right),\\ Z\left(t\right)=HX\left(t\right)+v\left(t\right), \end{array}\right. \end{array}$$

where *w*(*t*) denotes the system noise and *v*(*t*) is the observation noise. The above system state transition matrix coefficient *A* is

(14) $$\begin{array}{c} A=\left[\begin{array}{cccc} \Phi_{11} & 0 & \cdots & 0\\ \Phi_{21} & \Phi_{22} & \cdots & 0\\ \vdots & \vdots & \ddots & \vdots \\ \Phi_{n1} & \Phi_{n2} & \cdots & \Phi_{nn} \end{array}\right]. \end{array}$$

The noise covariance matrix *Q* of the state equation is written as

(15) $$\begin{array}{c} Q=\left[\begin{array}{cccc} \sigma_{\varepsilon_{1}}^{2} & 0 & \cdots & 0\\ 0 & \sigma_{\varepsilon_{2}}^{2} & \cdots & 0\\ \vdots & \vdots & \ddots & \vdots \\ 0 & 0 & \cdots & \sigma_{\varepsilon_{n}}^{2} \end{array}\right]. \end{array}$$

The observation matrix *H* is

(16) $$\begin{array}{c} H=\left[\begin{array}{cccc} \phi_{n1,} & \phi_{n2,} & \cdots & \phi_{nn} \end{array}\right]. \end{array}$$

The noise covariance matrix *R* of the observation equation is

(17) $$\begin{array}{c} R=\sigma_{\varepsilon_{n}}^{2}. \end{array}$$

Through the mentioned *A*, *H*, *Q*, and *R*, a complete state space model of SEMG can be determined. Based on the built system model, the digital filtering method is adopted to optimally estimate the signal sequence. To be specific, a Kalman filter refers to a recursive unbiased linear minimum variance estimation method, capable of estimating the current signal value by complying with the existing system estimation value and the current observation value.

As impacted by the time-varying and randomness of noise in practice, the statistical characteristics of noise may remain unknown and time-varying. Accordingly, the prior data commonly loses its meaning, causing the filtering effect to lose its optimality or to eventually lead to divergence [15].

To solve this type of problem, AKF is introduced. This method is capable of estimating the system's interference noise and measurement noise online based on the system measurement value and the filter value, tracking the noise change in real time while filtering, as well as correcting the filter parameters to increase the filtering accuracy [16]. Since the AKF algorithm is more sensitive to the initial value, a robust tracking AKF is introduced. The proposed method regulates the prediction error value by introducing a fading factor, i.e., to modify the filter gain matrix value, which increases the weight of the current observation. For this reason, the filter can track the current change and suppress the filter divergence [17].

Given the mentioned analysis, to optimize and improve the conventional Kalman filter algorithm, a strong tracking idea is introduced by using the simplified Sage-Husa adaptive filter algorithm. The improved strong tracking adaptive Kalman filter algorithm abides by the principle below:

(18) $$\begin{array}{c} \left\{\begin{array}{c} X\left(k\;|\;\;k-1\right)=A\left(k,k-1\right)X\left(k-1\right)+B\left(k,k-1\right)U\left(k-1\right)\\ V\left(k\right)=Z\left(k\right)-H\left(k\right)X\left(k\;\;|\;\;k-1\right)\\ P\left(k\;|\;k-1\right)=\lambda \left(k\right)A\left(k\;|\;k-1\right)P\left(k-1\right)A^{T}\left(k,k-1\right)+Q\left(k\right)\\ K\left(k\right)=P\left(k\;|\;k-1\right)H^{T}\left(k\right){\left[H\left(k\right)P\left(k\;|\;k-1\right)H^{T}\left(k\right)+R\left(k\right)\right]}^{-1}\\ X\left(k\right)=X\left(k\;|\;k-1\right)+K\left(k\right)V\left(k\right)\\ P\left(k\right)=\left[1-K\left(k\right)H\left(k\right)\right]P\left(k\;|\;k-1\right){\left[1-K\left(k\right)H\left(k\right)\right]}^{T}\\ +K\left(k\right)R\left(k-1\right)K^{T}\left(k\right) \end{array}\right), \end{array}$$

(19) $$\begin{array}{c} \left\{\begin{array}{c} Q\left(k\right)=\left(1-d_{k}\right)Q\left(k-1\right)+d_{k}\left[K\left(k-1\right)V\left(k\right)V{\left(k\right)}^{T}+\right]\\ A\left(k,k-1\right)P\left(k-1\right)A{\left(k,k-1\right)}^{T}\\ R\left(k\right)=d_{k}\left\{\left[1-H\left(k\right)K\left(k-1\right)\right]V\left(k\right)V^{T}\left(k\right){\left[1-H\left(k\right)K\left(k-1\right)\right]}^{T}+\right\}\\ H\left(k\right)P\left(k-1\right)H^{T}\left(k\right)+\left(1-d_{k}\right)R\left(k-1\right) \end{array}\right), \end{array}$$

(20) $$\begin{array}{c} \begin{array}{c} \lambda \left(k\right)=\left\{\begin{array}{c} \lambda_{0}\\ 1 \end{array}\right.\begin{array}{c} \;\lambda_{0}\geq 1\\ \lambda_{0}<1 \end{array}\\ \lambda_{0}=\frac{tr\left[N\left(k\right)\right]}{tr\left[M\left(k\right)\right]}\\ N\left(k\right)=V_{0}\left(k\right)-H\left(k\right)Q\left(k-1\right)H^{T}\left(k\right)-\beta R\left(k\right)\\ M\left(k\right)=H\left(k\right)A\left(k,k-1\right)P\left(k-1\right)A^{T}\left(k,k-1\right)H^{T}\left(k\right)\\ V_{0}\left(k\right)=\left\{\begin{array}{c} V\left(1\right)V^{T}\left(1\right)\\ \frac{\rho V_{0}\left(k\right)+V\left(k+1\right)V^{T}\left(k+1\right)}{1+\rho } \end{array}\right.\;\begin{array}{c} k=1\\ k>1 \end{array} \end{array}, \end{array}$$

where *d*_*k*_ = (1 − *b*)/(1 − *b*^*k*+1^), 0 < *b* < 1 and *b* is the forgetting factor, which usually refers to 0.95~0.99.

As presented above, equations (18), (19), and (20) constitute AKF, where equation (19) describes an adaptive noise statistical estimator, equation (18) is an optimal state estimator, and equation (20) expresses an adaptive fading factor. By alternately using the mentioned equations, an estimate of the state and noise statistics can be calculated. The initial conditions of *Q* and *R* can take the values of equations (15) and (17).

On the surface, under the unknown system noise variance matrix *Q* and the measurement noise variance matrix *R*, *Q* and *R* can be estimated simultaneously by the above process, which has been extensively investigated. As a matter of fact, the Sage-Husa method cannot estimate *Q* and *R* under the two unknown matrices. Filtering divergence is prone to occur under the high order of the system, and *Qk* and *Rk* are suggested to lose positive semidefiniteness and positive definiteness when filtering divergence. Thus, (19) is replaced with (21) only to iteratively update *Q* and fix *R*.

(21) $$\begin{array}{c} \left.\begin{array}{c} Q\left(k\right)=\left(1-d_{k}\right)Q\left(k-1\right)+d_{k}\left[K\left(k-1\right)V\left(k\right)V{\left(k\right)}^{T}+A\left(k,k-1\right)P\left(k-1\right)A{\left(k,k-1\right)}^{T}\right]\\ R\left(k\right)=R\left(0\right) \end{array}\right\}. \end{array}$$

In brief, the following sEMG denoising method is proposed based on the AR-AKF model.

According to Figure 1, the optimal order *n*∗ of the system is first determined by the information inspection criterion. Next, the autoregressive (AR) model is employed to express the sEMG signal fluctuation sequence, and the corresponding AR model group is built. Subsequently, the AR model group in the previous step is transformed into the state space model required for optimal estimation. Lastly, the AKF adaptive noise estimator is employed to adaptively estimate the statistical characteristics of the observed signal, and the optimal state estimator is adopted to optimally estimate the observed signal. To be specific, the state space model is the combination of AR and AKF, which also underpins AKF to perform filtering estimation.

## 3. Experiment Analysis

In the experiment here, the Trigno Wireless System of DELSYS is employed to collect EMG signals, and healthy men are taken as the experimental subjects. The collection frequency reaches 1000 Hz. The sEMG signals of the superficial flexor muscles of the fingers are collected to determine discrete sEMG sampling values. On the whole, 40 sets of wrist upturning are collected. There are 2000 data points per group. The Trigno sensor integrates a 20-450 Hz bandpass filter, so the frequency of the collected sEMG signal largely ranges from 20 to 450 Hz.

To verify the effectiveness of the denoising model proposed here, in the experiment, the standard sEMG signal is added with a SNR of 5 dB, 10 dB, 15 dB, 20 dB, 25 dB, and 30 dB band-limited Gaussian white noise, and the root mean square error (RMSE) and Mean Absolute Percentage Error (MAPE) are introduced, and also SNR is presented as an evaluation index. In addition to these evaluation indexes, a local similarity metric [18] is used for quantitative experimental results; it can reflect the signal leakage which refers to those lost coherent signal energy in the removed noise section. To compare the denoising effect of the denoising method proposed and the classic denoising method, simulation comparison experiments based on four denoising methods, i.e., AR-AKF, wavelet-sym8, LMS, and EMD, are designed.

Figure 2 illustrates a comparison diagram of the signal denoising effects exerted by the four methods (i.e., AR-AKF, wavelet-sym8, LMS, and EMD) under 5 dB of noisy signal.  Figure 3 shows the signal denoising error curve. Obviously, the sym8 wavelet method exerts a more significant denoising effect on low-amplitude signals, whereas it loses part of the real information in high-amplitude signals. According to Figure 2, the denoising result of EMD is suggested to be more effective than that of AR-AKF. However, as revealed by the data in Table 1, neither the mean RMSE nor the mean SNR is as good as AR-AKF. Through the combination of Figure 3, though most of the denoising error results of EMD are good, there is a period of very unsatisfactory results, and the final result is not as good as AR-AKF.

Table 1 presents the evaluated denoising effect of the four methods under a range of noise signals. Specific to low polluted signals, AR-AKF has the highest SNR and other methods have much lower SNR than the undenoised signal. For highly polluted signals, though the AR-AKF method does not make significant improvement compared to other methods, there are still more glitches in the denoised signal. The four methods are not extremely effective in denoising signals with low SNR ideally, and the advantage of AR-AKF indicates that it is capable of adaptively filtering and estimating the noise signal, so relatively ideal denoising results can be achieved in different noise levels.  Table 2 presents the local similarity metric of the four methods in different noise levels. In the original paper, the index of the local similarity metric is a map which has detailed information about the similarity between the original signal and denoised signal; for simplicity in this experiment, the local similarity metric is assigned the mean of all elements.  Table 2 indicates that AR-AKF has the best performance for low polluted signals which means that the lost coherent signal energy in the removed noise section is least; for highly polluted signals, AR-AKF is not the best but not badly performed compared to others. Generally speaking, the results of Table 2 are basically consistent with those of Table 1.

Overall, the AR-AKF method, as compared with other methods, is subject to a smaller root mean square error and a larger SNR, which also shows that the method based on the AR-AKF model exhibits a stronger denoising ability.

To more specifically study the effect of the AKF type in the overall model on the denoising effect, the four methods (i.e., AR-RTS, AR-SHKF, AR-STKF, and AR-STSHKF) are compared longitudinally. To be specific, RTS, SHKF, STKF, and STSHKF refer to a volumetric Kalman smoother, a Sage-Husa adaptive Kalman filter, a strong tracking adaptive filter, and a strong tracking adaptive filter based on Sage-Husa.

Figure 4 plots the signal denoising effect error curves of the four methods of AR-RTS, AR-SHKF, AR-STKF, and AR-STSHKF.  Table 3 lists the denoising evaluation results of the four methods. Obviously, the denoising effect achieved by different AKFs is different. To be specific, the optimal denoising effects are AR-STSHKF and AR-RTS. The average RMSE and SNR of AR-RTS are significantly better than those of other methods. AR-STSHKF is second only to AR-RTS. However, AR-RTS is primarily applied in offline scenarios, and AR-STSHKF can be exploited to achieve real-time online prediction. As a result, AR-STSHKF is more often employed in practice. Nevertheless, under weak real-time performance, the effect of the filter using the RTS smoother is more significant.

Moreover, the denoising effects under different orders are compared to determine the impact of the AR order on the denoising effect.  Figure 5 presents the size of the information criterion under different orders *n*.  Table 4 lists the AR-AKF denoising effect data table under different AR orders. To be specific in Figure 6, the AR-RTS denoising effect is optimal when *n* = 4, and the optimal denoising of the AR-STSHKF method is *n* = 3, basically consistent with the estimation of the information criterion.

## 4. Conclusion

In brief, a denoising method is developed in this study by employing the AR-AKF model based on the characteristics of the EMG signal. First, the optimal order *n* of the AR model is determined by abiding by the FPE, AIC, and BIC criteria of the Akaike information test. Subsequently, the AR model of this order is adopted to express the EMG signal sequence. Thus, *n* 1 to *n* orders are determined. The AR model equation set is used to build the state space model and the observation model by applying *n* AR model equation sets. Next, the adaptive Kalman filter method is adopted to obtain the optimal estimation of the original sEMG signal. As demonstrated from the experimental results, the model is capable of effectively removing the noise in the sEMG signal since the denoising effect of AKF complies with the accurate modeling of the target object. Accordingly, this study uses the AR model to build the precise mathematical model required for filtering the EMG signal sequence. Moreover, this mathematical model can describe the regular EMG signal and filter most irregular noises, so the model can be compared with reality. The signal data are fitted. Lastly, the dynamic modeling capabilities of AR and the characteristics of AKF's adaptive noise estimation are integrated, and the model parameters are regulated with the time-varying noise estimator to achieve a stable denoising effect, having strong adaptive capabilities and tracking performance.

In the experiment, the denoising effect of this model is compared with those of some classic methods, and the different effects exerted by different adaptive filters are analyzed in depth. As revealed from the experimental results, for the random noise of sEMG, the denoising effect of this model is significantly enhanced. Furthermore, the impact of different AR orders on the denoising results is experimentally analyzed, and the validity of the AR optimal order estimation criteria is verified.

## Figures and Tables

**Figure 1:** Denoising model based on AR-AKF.

**Figure 2:** Comparison chart of denoising effect.

**Figure 3:** Signal denoising error curve.

**Figure 4:** Signal denoising error comparison chart.

**Figure 5:** Different order information check criterion function value graph.

**Figure 6:** Comparison chart of denoising error under different orders.

**Table 1:** Signal denoising effect evaluation table.

Noisy signal (dB)	Sym8			EMD			LMS			AR-AKF		
	RMSE	SNR	MAPE	RMSE	SNR	MAPE	RMSE	SNR	MAPE	RMSE	SNR	MAPE
5	34.697	7.007	2.804	32.089	7.686	5.202	35.603	6.783	5.669	35.603	6.783	5.669
10	24.091	10.176	1.576	26.472	9.357	3.794	20.609	11.532	4.001	21.168	11.299	4.645
15	16.084	13.685	1.241	29.907	8.297	2.009	16.804	13.305	1.785	13.068	15.488	2.031
20	10.757	17.179	0.886	30.595	8.100	1.488	15.558	13.974	1.475	7.735	20.043	1.374
25	7.447	20.373	0.700	36.225	6.633	1.052	14.981	14.302	0.913	4.569	24.615	0.761
30	5.548	22.930	0.581	38.624	6.076	1.151	14.723	14.456	0.947	2.960	28.385	0.619

**Table 2:** Local similarity metric evaluation table.

Noisy signal (dB)	Sym8	EMD	LMS	AR-AKF
	Mean of local similarity metric			
5	0.6280	0.7061	0.6683	0.6465
10	0.7301	0.7917	0.7737	0.7448
15	0.8332	0.8300	0.8511	0.8310
20	0.8512	0.8240	0.8831	0.8758
25	0.8676	0.8699	0.9004	0.9026
30	0.8895	0.8450	0.9092	0.9175

**Table 3:** Nonnoise effect data statistics table.

	AR-RTS	AR-SHKF	AR-STKF	AR-STSHKF
RMSE	29.7808	33.1007	32.7497	32.5449
SNR	8.3347	7.4167	7.5093	7.5638

**Table 4:** Data table of denoising effect under different orders.

*n*	RMSE	
	AR-RTS	AR-STSHKF
*n* = 2	25.9384	26.8722
*n* = 3	25.5518	26.8495
*n* = 4	25.2164	26.8683
*n* = 5	25.8643	26.8719
*n* = 6	25.9564	26.8689

## Data Availability

No data, models, or code were generated or used during the study.
